This article has been retracted.

# Causal effects of omega‐6 and LDL‐C on androgenetic alopecia: A Mendelian randomization study

**DOI:** 10.1111/srt.70000

**Published:** 2024-08-13

**Authors:** Liu Peilong, Zhao Quanlin, Gu Shuqing

**Affiliations:** ^1^ The First Clinical Medical College Shandong University of Traditional Chinese Medicine Jinan Shandong China; ^2^ General Internal Medicine Affiliated Hospital of Shandong University of Traditional Chinese Medicine Jinan Shandong China; ^3^ Internal Medicine People's Hospital of Xiajin County Xiajin China

**Keywords:** androgenic alopecia, LDL‐C, Mendelian randomization, Omega‐6

## Abstract

**Background:**

Increasing studies have reported a causal relationship between androgenetic alopecia (AGA) and lipid‐related metabolites. However, the relationships between HDL‐C, LDL‐C, Omega‐6, and Omega‐3 with AGA remain unclear. Some research findings are even contradictory. Therefore, we designed this study to explore this issue.

**Methods:**

In this study, we selected seven exposure factors, screened SNPs with significant associations, removed linkage disequilibrium and weak instrumental variables, and conducted bidirectional MR analysis.

**Results:**

The study found that omega‐6 and LDL‐C, especially total cholesterol in medium LDL and total cholesterol in small LDL, are risk factors for the occurrence of androgenetic alopecia.

**Conclusion:**

In summary, we found that various lipid‐related metabolites have a causal relationship with the occurrence of androgenetic alopecia, providing new insights into the pathogenesis of androgenetic alopecia and offering references for clinical treatment of androgenetic alopecia.

## 1 INTRODUCTION

Androgenetic alopecia is a common clinical condition, with more than 80 out of every 100 men over the age of 70 suffering from it as they age.^1^ The incidence in women is lower than in men. Due to the complexity of its etiology, treatment options for androgenetic alopecia are still being refined. Currently, finasteride is the only oral medication widely approved by various countries for the treatment of androgenetic alopecia. Clinically, it can be challenging to accurately diagnose androgenetic alopecia, requiring doctors to combine family history, laboratory results, and clinical symptoms for a comprehensive judgment.^2^ Once a patient is suspected of having androgenetic alopecia, the evaluator generally needs to comprehensively assess whether the patient's scalp hair follicles show inflammatory reactions and whether the hair loss areas conform to androgenetic alopecia characteristics. Sometimes, the pull test is also an important diagnostic method; if more than six hairs are pulled out in a single area, it is considered abnormal hair shedding.^3^ In recent years, the global demand for safe and natural hair loss treatment products has been increasing, with a market value reaching 3 billion USD in 2017 and expected to grow by approximately 4% by 2024.^4^ The application of nutritional supplements has gradually attracted the attention of the scientific community and the market. A survey shows that 75% of dermatologists occasionally use dietary supplements, with more than 25% using Omega‐3 fatty acids.^5^

Some studies have shown that multiple lipid metabolism abnormalities have been found in patients with AGA. These include HDL, LDL, and serum lipid metabolites such as phosphatidylcholine (PC) and lysophosphatidylcholine (LPC),^6^ a Mendelian randomization (MR) study analyzed the causal relationship of LDL, HDL, VLDL, Apolipoprotein A1, Apolipoprotein B, total cholesterol, polyunsaturated fatty acid, Omega‐3, and Omega‐6 particle concentrations with AGA. Apolipoprotein B, LDL, and VLDL were found to be risk factors for AGA,^7^ guiding us to further clarify the research direction. However, the relationship between various lipid metabolism products, including Omega‐3, Omega‐6, HDL‐C, and LDL‐C, and AGA, remains unclear. These substances are integral to the ongoing research and market focus on the “relationship between nutritional supplements and AGA.” In particular, various natural oil‐based nutritional supplements, such as fish oil, are rich in Omega‐3 and contain relatively smaller amounts of Omega‐6. It remains to be determined through more rigorous research whether these supplements have potential protective effects or pose risks for AGA.

We used the latest genome‐wide association study (GWAS) data to investigate the levels of Omega‐3, Omega‐6, HDL‐C, LDL‐C, total cholesterol in medium LDL, and total cholesterol in small LDL as our main research direction. Current studies have confirmed that lipids‐related metabolites (LRMs) are highly heritable,^8^ and AGA also has a causal relationship with genetic factors, providing a basis for using the mendelian randomization research method.^9^ In this research, we used the latest genome‐wide association study results. This study included up to 136 016 participants from 33 cohorts with quantification of the characteristics of 233 circulating metabolites using nuclear magnetic resonance (NMR) spectroscopy, and manually curated potential candidate genes, assigning possible pathogenic genes in two‐thirds of the loci. This study included over six times more participants than the largest GWAS of circulating metabolites based on mass spectrometry, thus allowing a deeper characterization of genetic regulation.^10^ Compared with previous GWAS meta‐analyses of NMR metabolic traits, the sample size increased fivefold and the number of metabolic traits doubled,^11^ greatly improved understanding of the genetic basis of metabolism.^12^ The use of bidirectional MR studies can evaluate the effects of genetically predicted exposure factors on disease and the reverse causal relationship of the disease on exposure factors. This method provides more comprehensive causal inference capabilities, helping to determine the complex relationships between variables.^13^

## 2 MATERIALS AND METHODS

### 2.1 Study design of Mendelian randomization

As shown in Figure 1, we used a bidirectional MR approach to study the problem. This method reduces confounding factors and eliminates reverse causation interference during the study. In this process, we are based on three core assumptions of MR: (1) Relevance needs to be satisfied. The genetic variation used as an instrumental variable must be closely related to the exposure factor. (2) Independence needs to be satisfied. The genetic variation used as an instrumental variable cannot be related to any potential confounding factors. (3) Exclusion needs to be satisfied. The genetic variation used as an instrumental variable can and can only be related to the outcome variable through the exposure factor.^14^, ^15^

**FIGURE 1:** The flow chart delineates the assumptions and methodological details of the bidirectional Mendelian randomization employed in this study, encompassing data sources, exposure variables, outcome measures, and analytical techniques.

### 2.2 GWAS data sources

The exposure data are from the study by Karjalainen et al. The complete data set is available at the public URL https://www.phpc.cam.ac.uk/ceu/

Data on androgenic alopecia are from Finn Gen Biobank and can be accessed by visiting https://gwas.mrcieu.ac.uk/

### 2.3 Selection criteria of instrumental variables for LRMs

In this study, we initially set *p* < 5e−8 to select single SNPs. However, the significant SNPs available for exposure assessment were limited, so we applied a *p*‐value threshold of *p* < 1e‐5 to expand the search range. We set *r* ^2^ < 0.001 and a threshold of 10 000 kb to remove linkage disequilibrium, ensuring genetic independence.^16^ We calculated an *F*‐statistic threshold of 10, and SNPs with *F*‐statistics below this value were excluded to eliminate weak instrumental variables.^17^

### 2.4 MR STATISTICAL ANALYSIS

The causal effects between LRMs and AGA were primarily evaluated using inverse variance weighting, Mr‐Egger method, weighted median method, simple mode, and weighted mode. The final results were analyzed mainly using the IVW method, with a *p*‐value < 0.05 considered significant. All conclusions required testing for pleiotropy to ensure that pleiotropic effects could be considered negligible. A leave‐one‐out test was used to sequentially remove SNPs and check the impact on the remaining results to ensure causal relationships and reliability. Finally, to test whether there was a reverse causal relationship between the outcome and the exposure we studied, we treated the SNPs associated with AGA with the same criteria, swapped the exposure and outcome, and performed a reverse MR analysis. The main tool used in the MR analysis was TwoSampleMR version 0.6.4.

## 3 RESULTS

In the two‐sample MR analysis, four types of LRMs were ultimately considered risk factors for the occurrence of AGA, including the OR of Omega‐6 fatty acids levels by IVW method was 1.615687857 (95% CI: 1.024342513–2.5484124873, *p* = 0.03907053). The OR of Total cholesterol levels in LDL by IVW method was 1.543318598 (95% CI: 1.036756749–2.297387787, *p* = 0.032529872). The OR of Total cholesterol levels in medium LDL by IVW method was 1.564847429 (95% CI: 1.026767417–2.384909607, *p* = 0.037263038). The OR of Total cholesterol levels in small LDL by IVW method was 1.56595347 (95% CI: 1.053814469–2.326984817, *p* = 0.026460656). Other exposures, including serum HDL‐C, Total cholesterol in large LDL, and Omega‐3 fatty acids levels, did not show reliable causal relationships with AGA in the analysis. (See Table 1 for all analysis data and Figure 2 for the visualized results). None of the positive results demonstrated pleiotropy, as shown in Table 2. Figure 3 shows the trend of the relationship between exposure and outcome under different analysis methods. Figure 4 shows the heterogeneity of SNPs. If there are particularly outliers, it means heterogeneity may exist. The results of the leave‐one‐out test are shown in Figure 5. Meanwhile, the reverse MR analysis did not yield any positive conclusions, indicating that AGA did not significantly affect the selected LRMs.

**TABLE 1:** MR analysis results of seven exposure instrumental variables.

	Method	nsnp	or	or_lci95	or_uci95	pval
Omega‐6 fatty acids levels	MR Egger	158	1.744820693	0.823393685	3.697379888	0.148278758
	Weighted median	158	1.374756153	0.660533143	2.861256093	0.39472994
	Inverse variance weighted	158	1.615687857	1.024342513	2.548412487	0.039070583
	Simple mode	158	3.154458249	0.815002315	12.20929887	0.098158191
	Weighted mode	158	1.333271147	0.664653118	2.674495766	0.419245335
Total cholesterol levels in LDL	MR Egger	156	1.502973507	0.858172602	2.63225528	0.156165493
	Weighted median	156	0.912818335	0.495584419	1.681322658	0.769742541
	Inverse variance weighted	156	1.543318598	1.036756749	2.297387787	0.032529872
	Simple mode	156	1.099395474	0.302857405	3.9908894	0.885639843
	Weighted mode	156	1.246933313	0.713193224	2.180114216	0.439982302
Total cholesterol in medium LDL	MR Egger	152	1.596927623	0.886161155	2.87778111	0.121391176
	Weighted median	152	0.953694195	0.501521124	1.81354797	0.885034198
	Inverse variance weighted	152	1.564847429	1.026767417	2.384909607	0.037263038
	Simple mode	152	1.179405843	0.334278955	4.161189697	0.797896527
	Weighted mode	152	1.259341787	0.752935256	2.10634543	0.380978888
Total cholesterol in small LDL	MR Egger	158	1.540373957	0.883316621	2.68618508	0.129857922
	Weighted median	158	0.95085793	0.50390751	1.794239585	0.876393041
	Inverse variance weighted	158	1.56595347	1.053814469	2.326984817	0.026460656
	Simple mode	158	1.03528538	0.287291542	3.730760091	0.957784018
	Weighted mode	158	1.250410159	0.714865878	2.187159318	0.434592955
Total cholesterol levels in HDL	MR Egger	178	0.523316728	0.249186989	1.099015637	0.088917623
	Weighted median	178	0.610500855	0.304840804	1.222642403	0.163712308
	Inverse variance weighted	178	0.679705802	0.439939293	1.050144838	0.081937329
	Simple mode	178	0.890481577	0.220400208	3.597807117	0.870847242
	Weighted mode	178	0.542953182	0.275541653	1.069886002	0.079322309
Total cholesterol in large LDL	MR Egger	163	1.458266678	0.820657282	2.591266476	0.2002362
	Weighted median	163	0.916954182	0.479705299	1.752753145	0.793105326
	Inverse variance weighted	163	1.472225729	0.982382731	2.206317893	0.060946221
	Simple mode	163	1.0633557	0.259325727	4.360251314	0.932108361
	Weighted mode	163	1.271258395	0.747604373	2.16170205	0.376883332
Omega‐3 fatty acids levels	MR Egger	112	1.162869918	0.583232421	2.318572147	0.669066721
	Weighted median	112	0.845116432	0.406296598	1.757882758	0.652459832
	Inverse variance weighted	112	0.994845099	0.624215235	1.585537672	0.982660659
	Simple mode	112	0.623625822	0.157955282	2.46214727	0.501731642
	Weighted mode	112	0.876332897	0.459793938	1.670225036	0.68907023

**FIGURE 2:** MR analysis results and forest plot of seven substances.

**FIGURE 3:** The trend of the relationship between exposure and outcome under different analysis methods.

**TABLE 2:** The results of pleiotropy testing.

	egger_intercept	se	pval
Omega‐6 fatty acids levels	−0.004570459	0.018070432	0.800659385
Total cholesterol levels in LDL	0.002025088	0.015344075	0.895173551
Total cholesterol in medium LDL	−0.001535046	0.015824307	0.922851437
Total Cholesterol in small LDL	0.001224056	0.014752847	0.933981081

**FIGURE 4:** The heterogeneity of SNPs. If there are particularly outliers, it means heterogeneity may exist.

**FIGURE 5:** A leave‐one‐out graph showing the impact of removing each SNP on the overall analysis results.

## 4 DISCUSSION

Androgenic alopecia is the most common form of hair loss, and it generally begins gradually after puberty.^1^ Increased androgen levels in hair follicles and sensitivity to androgens are considered the most important factors leading to AGA.^18^ Studies have shown that the incidence of AGA is lower in people who have had their testicles removed before puberty and in people with complete androgen insensitivity syndrome, which supports the view that androgens are an important factor in the occurrence of AGA.^19^

Studies on the association between LDL‐C and androgens have reported that testosterone may have an inhibitory effect on LDL‐C,^20^ which can lead to unclear directions of causality in observational studies. Our study used Mendelian randomization analysis to indirectly measure exposure through genetic variation, ensuring clarity in the direction of causality. The results showed that LDL‐C, total cholesterol in medium LDL, and total cholesterol in small LDL had a positive causal relationship with the occurrence of AGA. This phenomenon may be related to the mediating effects of androgens and inflammatory factors. Research indicates that cholesterol is the fundamental precursor of steroid hormones (such as testosterone and dihydrotestosterone). LDL‐C binds to LDL receptors on the cell surface, is internalized by the cells, releases cholesterol, and transports cholesterol in the blood, delivering it to cells that need to synthesize steroid hormones, particularly Leydig cells in the testes.^21^, ^22^ Metabolic diseases such as hypercholesterolemia or hypocholesterolemia may affect androgen production by altering LDL‐C levels. For example, abnormal LDL receptor function or LDL‐C metabolic disorders may lead to abnormal androgen levels.^21^ LDL‐C has been shown to induce a stronger inflammatory response. LDL‐C is prone to oxidation, forming oxidized low‐density lipoprotein, which then stimulates the release of inflammatory factors such as interleukins.^23^ In the scalp tissues of AGA patients, the levels of these inflammatory factors are often elevated, leading to increased inflammation around hair follicles, damaging follicular structures, and impairing normal follicular function.^24^, ^25^

Omega‐6 also has a complex relationship with androgen levels. Omega‐6 can inhibit the kisspeptin‐GnRH signaling pathway. This reduces the production of luteinizing hormone, follicle‐stimulating hormone, and testosterone, and can also inhibit the mRNA expression of some steroidogenic genes, such as CYP17A1, CYP19. It can also promote androgen synthesis by increasing precursor products.^26^, ^27^ Some observational studies suggest that Omega‐6 can reduce the occurrence of AGA. Omega‐6 contains gamma‐linolenic acid, which can reduce the production of dihydrotestosterone. Dihydrotestosterone is an important cause of AGA. Omega‐6 may reduce the risk of AGA by inhibiting it.^28^ However, previous research is limited by insufficient sample sizes and has not reached sufficiently strong conclusions. This study found that omega‐6 is a risk factor for the occurrence of AGA. It is speculated that the mechanism may be related to promoting the synthesis of steroid hormones. Highly unsaturated Omega‐6 fatty acids (such as arachidonic acid, ARA) preferentially serve as substrates for hormone‐sensitive lipase (HSL), increasing the release of free cholesterol and thereby promoting the synthesis of steroid hormones. Leydig cells highly express the enzyme FADS2, which is critical for the biosynthesis of highly unsaturated fatty acids (HUFAs). By inhibiting FADS2, the level of omega‐6 in Leydig cells can be reduced, thereby inhibiting the production of androgens. At the same time, if omega‐6 is supplemented, the production capacity of androgens can be restored. This experiment shows that omega‐6 plays an important role in the production of androgens and may therefore increase the risk of AGA.^29^

This study found that the level of omega‐6 and the level of LDL‐C are risk factors for the occurrence of AGA. This not only provides a reference for further research on the effects of unsaturated fatty acids on AGA, but also suggests that nutritional supplements currently being explored for AGA treatment, such as pumpkin seed oil,^30^ which is rich in Omega‐6, may pose potential risks. Future research should more cautiously evaluate the effects of these complex natural nutritional supplements.

Many studies have reported the therapeutic effects of Omega‐3 on AGA,^31^, ^32^ but this study did not find a significant causal relationship between Omega‐3 and AGA. The limited sample size and the potential heterogeneity between the mechanisms of therapeutic and preventive effects may explain this discrepancy, which does not necessarily contradict the findings of other studies on Omega‐3′s therapeutic effects. Further research is needed to elucidate the mechanism of Omega‐3′s therapeutic effects and its clinical efficacy.

However, our study has some limitations. First, we are still unclear through which mediators Omega‐6 and LDL‐C affect the onset of AGA. Second, the data used in our study came from a European population, which may limit the applicability of our findings to other demographic groups. In conclusion, our study reveals the causal effects of Omega‐6 and LDL‐C on AGA through MR analysis. Considering the results of sensitivity analyses, our findings are reliable. Our findings do not negate the possibility of non‐genetic associations. Conducting broader studies is crucial for exploring these potential connections.

## CONFLICT OF INTEREST STATEMENT

The authors declare no conflicts of interest.

## ETHICS STATEMENT

The GWAS data used in this study were public de‐identified data. There was no need for additional ethical approval.

## Data Availability

The data that support the findings of this study are available from the corresponding author upon reasonable request.
